# Classification of Breast Cancer Histopathological Images Using DenseNet and Transfer Learning

**DOI:** 10.1155/2022/8904768

**Published:** 2022-10-10

**Authors:** Musa Adamu Wakili, Harisu Abdullahi Shehu, Md. Haidar Sharif, Md. Haris Uddin Sharif, Abubakar Umar, Huseyin Kusetogullari, Ibrahim Furkan Ince, Sahin Uyaver

**Affiliations:** ^1^Abubakar Tafawa Balewa University, Bauchi 740272, Nigeria; ^2^School of Engineering and Computer Science, Victoria University of Wellington, Wellington 6012, New Zealand; ^3^College of Computer Science and Engineering, University of Hail, Hail 2440, Saudi Arabia; ^4^School of Computer & Information Sciences, University of the Cumberlands, Williamsburg, KY 40769, USA; ^5^Department of Computer Science, Blekinge Institute of Technology, Karlskrona 37141, Sweden; ^6^Department of Digital Game Design, Nisantasi University, 34485 Istanbul, Turkey; ^7^Department of Energy Science and Technologies, Turkish-German University, 34820 Istanbul, Turkey

## Abstract

Breast cancer is one of the most common invading cancers in women. Analyzing breast cancer is nontrivial and may lead to disagreements among experts. Although deep learning methods achieved an excellent performance in classification tasks including breast cancer histopathological images, the existing state-of-the-art methods are computationally expensive and may overfit due to extracting features from in-distribution images. In this paper, our contribution is mainly twofold. First, we perform a short survey on deep-learning-based models for classifying histopathological images to investigate the most popular and optimized training-testing ratios. Our findings reveal that the most popular training-testing ratio for histopathological image classification is 70%: 30%, whereas the best performance (e.g., accuracy) is achieved by using the training-testing ratio of 80%: 20% on an identical dataset. Second, we propose a method named DenTnet to classify breast cancer histopathological images chiefly. DenTnet utilizes the principle of transfer learning to solve the problem of extracting features from the same distribution using DenseNet as a backbone model. The proposed DenTnet method is shown to be superior in comparison to a number of leading deep learning methods in terms of detection accuracy (up to 99.28% on BreaKHis dataset deeming training-testing ratio of 80%: 20%) with good generalization ability and computational speed. The limitation of existing methods including the requirement of high computation and utilization of the same feature distribution is mitigated by dint of the DenTnet.

## 1. Introduction

Breast cancer is one of the most familiar invasive cancers in women worldwide. Nowadays, it is overtaking lung cancer as the world's chiefly regularly diagnosed cancer [1]. The diagnosis of breast cancer in the early stages significantly decreases the mortality rate by allowing the choice of adequate treatment. With the onset of pattern recognition and machine learning, a good deal of handcrafted or engineered features-based studies have been proposed for classifying breast cancer histology images. In image classification, feature extraction is a cardinal process used to maximize the classification accuracy by minimizing the number of selected features [2–5]. Deep learning models have the power to automatically extract features, retrieve information, and take in the latest intellectual depictions of data. Thus, they can solve the problems of common feature extraction methods. The automated classification of breast cancer histopathological images is one of the important tasks in CAD (Computer-Aided Detection/Diagnosis) systems, and deep learning models play a remarkable role by detecting, classifying, and segmenting prime breast cancer histopathological images. Many researchers worldwide have invested appreciable efforts in developing robust computer-aided tools for the classification of breast cancer histopathological images using deep learning. At present, in this research arena, the most popular deep learning models proposed in the literature are based on CNNs [6–66].

A pretrained CNN model, for example, DenseNet [67], utilizes dense connection between layers, reduces the number of parameters, strengthens propagation, and encourages feature reutilization. This improved parameter efficiency makes the network faster and easier to train. Nevertheless, a DenseNet [67] has an excessive connection, as all its layers have a direct connection to each other. Those lavish connections have been shown to decrease the computational and parameter efficiency of the network. In addition, features extracted by a neural network model stay in the same distribution. Therefore, the model might overfit as the features cannot be guaranteed to be sufficient enough. Besides, a CNN-training task demands a large number of training samples; otherwise, it leads to overfitting and reduces generalization ability. However, it is arduous to secure labeled breast cancer histopathological images, which severely limits the classification ability of CNN [27].

On the other hand, the use of transfer learning can expand prior knowledge about data by including information from a different domain to target future data [68]. Consequently, it is a good idea to extract data from a related domain and then transfer those extracted data to the target domain. This way, resources can be saved and the efficiency of the model can be improved during training. A great number of breast cancer diagnosis methods based on transfer learning have been proposed and implemented by distinct researchers (e.g., [57–66]) to achieve state-of-the-art performance (e.g., ACC, AUC, PRS, RES, and F1S) on different datasets. Yet, the limitations of such performance indices, algorithmic assumptions, and computational complexities are indicating a further development of smart algorithms.

In this paper, we aim to propose a novel neural-network-based approach called DenTnet (see Figure 1) for classifying breast cancer histopathological images by taking the benefits of both DenseNet [67] and transfer learning [68]. To address the cross-domain learning problems, we employ the principle of transfer learning for transferring information from a related domain to the target domain. Our proposed DenTnet is anticipated to increase the accuracy of breast cancer histopathological images classification and accelerate the learning process. The DenTnet demonstrates better performance over its alternative CNN and/or transfer-learning-based methods (e.g., see Table 1) on the same dataset as well as training-testing ratio.

To find the best performance scores of deep learning models for classifying histopathological images, contrasting training-testing ratios were applied for divergent models on the same dataset. What would be the most popular and/or optimized training-testing ratios to classify histopathological images considering existing state-of-the-art deep learning models? There exist many surveys enriched to sufficient contemporary methods and materials with systematic deep discussion of automatic classification of breast cancer histopathological images [68–72]. Nevertheless, to the best of our knowledge, the direct or indirect indication of this question was not reported in any of the previous studies. Henceforth, we perform a succinct survey to investigate this question. Our findings include that the most popular training-testing ratio for histopathological image classification is 70%: 30%, whereas the best performance (accuracy) is achieved by using the training-testing ratio of 80%: 20% on the identical dataset.

In summary, the main contributions of this context are as follows:

- Determine the most popular and/or optimized training-testing ratios for classifying histopathological images using the existing state-of-the-art deep learning models.
- Propose a novel approach named DenTnet that amalgamates both DenseNet [67] and transfer learning technique to classify breast cancer histopathological images. DenTnet is anticipated to achieve high accuracy and fasten the learning process due to its utilization of dense connections from its backbone architecture (i.e., DenseNet [67]).
- Determine the generalization ability of DenTnet and the superiority measure considering nonparametric statistical tests.

The rest of the paper is organized as follows: Section 2 hints some preliminaries; Section 3 surveys briefly the existing deep models for histopathological image classification and reports our findings; Section 4 depicts the architecture of our proposed DenTnet and its implementation details; Section 5 demonstrates the experimental results and comparison on BreaKHis dataset [33]; Section 6 evaluates the generalization ability of DenTnet; Section 7 discusses nonparametric statistical tests, their reported results, and reasons for superiority along with few hints of further study; and Section 8 concludes the paper.

## 2. Preliminaries

Breast cancer is one of the oldest known kinds of cancer first found in Egypt [73]. It is caused by the uncontrolled growth and division of cells in the breast, whereby a mass of tissue called a tumor is created. Nowadays, it is one of the most terrifying cancers in women worldwide. For example, in 2020, there were 2.3 million women diagnosed with breast cancer and 685000 deaths globally [74]. Early detection of breast cancer can save many lives. Breast cancer can be diagnosed in view of histology and radiology images. The radiology images analysis can help to identify the areas, where the abnormality is located. However, they cannot be used to determine whether the area is cancerous [75]. On the other hand, a biopsy is an examination of tissue removed from a living body to discover the presence, cause, or extent of a disease (e.g., cancer). Biopsy is the only reliable way to make sure if an area is cancerous [76]. Upon completion of the biopsy, the diagnosis will be based on the qualification of the histopathologists who determine cancerous regions and malignancy degree [7, 75]. If the histopathologists are not well trained, the histopathology or biopsy report can lead to an incorrect diagnosis. Besides, there might be a lack of specialists, which may cause keeping the tissue samples for up to a few months. In addition, diagnoses made by unspecialized histopathologists are sometimes difficult to replicate. As if that were not enough of a problem, at times, even expert histopathologists tend to disagree with each other. Despite notable progress being reached by diagnostic imaging technologies, the final breast cancer grading and staging are still done by pathologists using visual inspection of histological samples under microscopes.

As analyzing breast cancer is nontrivial and would get down to disagreements among experts, computerized and interdisciplinary systems can improve the accuracy of diagnostic results by reducing the processing time. The CAD can help to assist doctors in reading and interpreting medical images by locating and identifying possible abnormalities in the image [69]. It is proclaimed that the utilization of CAD to automatically classify histopathological images does not only improve the diagnostic efficiency with low cost but also provide doctors with more objective and accurate diagnosis results [77]. Consequently, there is an adamant demand for the CAD [78]. There exist several comprehensive surveys for CAD based methods in the literature. For example, Zebari et al. [71] provided a common description and analysis of existing CAD systems that are utilized in both machine learning and deep learning methods as well as their current state based on mammogram image modalities and classification methods. However, the existing breast cancer diagnosis models take issue with complexity, cost, human-dependency, and inaccuracy [73]. Furthermore, the limitation of datasets is another practical problem in this arena of research. In addition, every deep learning model demands a metric to judge its performance. Explicitly, performance evaluation metrics are the part and parcel of every deep learning model as they indicate progress indices.

In the two following subsections, we discuss the commonly used datasets for classifying histopathological images and the performance evaluation metrics of various deep learning models.

### 2.1. Brief Description of Datasets

Accessing relevant images and datasets is one of the key challenges for image analysis researchers. Datasets and benchmarks enable validating and comparing methods for developing smarter algorithms. Recently, several datasets of breast cancer histopathology images have been released for this purpose.  Figure 2 shows a sample breast cancer histopathological image from BreaKHis [33] dataset of a patient who suffered from papillary carcinoma (malignant) with four magnification levels: (a) 40x, (b) 100x (c) 200x, and (d) 400x [79]. The following list of datasets has been used in the literature as incorporated in Table 2:

- BreaKHis [33] ⇒ It is considered as the most popular and clinical valued public breast cancer histopathological dataset. It consists of 7909 breast cancer histopathology images, 2480 benign and 5429 malignant samples, from 82 patients with different magnification factors (e.g., 40x, 100x, 200x, and 400x) [33].
- Bioimaging2015 [122] ⇒ The Bioimaging2015 [122] dataset contained 249 microscopy training images and 36 microscopy testing images in total, equally distributed among the four classes.
- ICIAR2018 [78] ⇒ This dataset, available as part of the BACH grand challenge [78], was an extended version of the Bioimaging2015 dataset [8, 122]. It contained 100 images in each of four categories (i.e., normal, benign, in situ carcinoma, and invasive carcinoma) [8].
- BACH [78] ⇒ The database of BACH holds images obtained from ICIAR2018 Grand Challenge [78]. It consists of 400 images with equal distribution of normal (100), benign (100), in situ carcinoma (100), and invasive carcinoma (100). The high-resolution images are digitized with the same conditions and magnification factor of 200x. In this dataset, images have a fixed size of 2048 × 1536 pixels [175].
- TMA [99] ⇒ The TMA (Tissue MicroArray) database from Stanford University is a public resource with an access to 205161 images. All the whole-slide images have been scanned by a 20x magnification factor for the tissue and 40x for the cells [176].
- Camelyon [97] ⇒ The Camelyon (cancer metastases in lymph nodes) was established based on a research challenge dataset competition in 2016. The Camelyon organizers trained CNNs on smaller datasets for classifying breast cancer in lymph nodes and prostate cancer biopsies. The training dataset consists of 270 whole-slide images; among them 160 are normal slides and 110 slides contain metastases [97].
- PCam [121] ⇒ It is a modified version of the Patch Camelyon (PCam) dataset, which consists of 327680 microscopy images with 96 × 96-pixel sized patches extracted from the whole-slide images with a binary label hinting the presence of metastatic tissue [8].
- HASHI [129] ⇒ Each image in the dataset of HASHI (high-throughput adaptive sampling for whole-slide histopathology image analysis) [129] has the size of 3002 × 2384 [161].
- MIAS [85] ⇒ The Mammographic Image Analysis Society (MIAS) database of digital mammograms [85] contains 322 mammogram images, each of which has a size of 1024 × 1024 pixels with PGM format [59].
- INbreast [92] ⇒ The INbreast database has a total of 410 images collected from 115 cases (i.e., patients) indicating benign, malignant, and normal cases having sizes of 2560 × 3328 or 3328 × 4084 pixels. It contains 36 benign and 76 malignant masses [92].
- DDSM [84] ⇒ The DDSM [84] dataset was collected by the expert team at the University of South Florida [84]. It contains 2620 scanned film mammography studies. Explicitly, it involves 2620 breast cases (i.e., patients) categorized in 43 different volumes with average size of 3000 × 4800 pixels [48].
- CBIS-DDSM [128] ⇒ The CBIS-DDSM [128] is an updated version of the DDSM providing easily accessible data and improved region-of-interest segmentation [128, 146]. The CBIS-DDSM dataset comprises 2781 mammograms in the PNG format [49].
- CMTHis [37] ⇒ The CMTHis (Canine Mammary Tumor Histopathological Image) [37] dataset comprises 352 images acquired from 44 clinical cases of canine mammary tumors.
- FABCD [133] ⇒ The FABCD (Fully Annotated Breast Cancer Database) [133] consists of 21 annotated images of carcinomas and 19 images of benign tissue taken from 21 patients [130].
- IICBU2008 [87] ⇒ The IICBU2008 (Image Informatics and Computational Biology Unit) malignant lymphoma dataset contains 374 H&E stained microscopy images captured using bright field microscopy [21].
- VLAD [136] ⇒ The VLAD (Vector of Locally Aggregated Descriptors) dataset [136] consists of 300 annotated images with resolution of 1280 × 960 [29].
- LSC [137] ⇒ The LSC (Lymphoma Subtype Classification) [137] dataset has been prepared by pathologists from different laboratories to create a real-world type cohort which contains a larger degree of stain and scanning variances [137]. It consists of 374 images with resolution of 1388 × 1040 [29].
- KimiaPath24 [126] ⇒ The official KimiaPath24 [126] dataset consists of a total of 23916 images for training and 1325 images for testing. It is publicly available. It shows various body parts with texture patterns [41].

### 2.2. Performance Evaluation Metrics

Performance evaluation of any deep learning model is an important task. An algorithm may give very pleasing results when evaluated using a metric (e.g., *ACC*), but it may give poor results when evaluated against other metrics (e.g., *F1S*) [177]. Usually, we use classification accuracy to measure the performance of deep learning algorithms. But it is not enough to determine the model perfectly. For truly judge any deep learning algorithm, we can use nonidentical types of evaluation metrics including classification *ACC*, *AUC*, *PRS*, *RES*, *F1S*, *RTM*, and *GMN*.

(i) ACC ⇒ It is normally defined in terms of error or inaccuracy [178]. It can be calculated using the following equation:
  (1) $$\begin{array}{c} ACC=\frac{\left(100\right)\left(t_{n}+t_{p}\right)}{t_{p}+t_{n}+f_{p}+f_{n}}\text{,} \end{array}$$
where *t*_*n*_ is true negative, *t*_*p*_ is true positive, *f*_*p*_ is false positive, and *f*_*n*_ is false negative. Sometimes, ACC and the percent correct classification (PCC) can be used interchangeably.
(ii) PRS ⇒ Its best value is 100 and the worst value is just 0. It can be formulated using the following equation:
  (2) $$\begin{array}{c} PRS=\frac{\left(100\right)\left(t_{p}\right)}{t_{p}+f_{p}}\text{.} \end{array}$$
(iii) RES ⇒ It should ideally be 100 (the highest) for a good classifier. It can be calculated using the following equation:
  (3) $$\begin{array}{c} RES=\frac{\left(100\right)\left(t_{p}\right)}{t_{p}+f_{n}}\text{.} \end{array}$$
(iv) AUC ⇒ It is one of the most widely used metrics for evaluation [177–179]. The *AUC* of a classifier equals the probability that the classifier ranks a randomly chosen positive sample higher than a randomly chosen negative sample. The *AUC* varies in value from 0 to 1. If the predictions of a model are 100% wrong, then its *AUC* = 0.00; but if its predictions are 100% correct, then its *AUC* = 1.00.
(v) F1S ⇒ It is the harmonic mean between precision and recall. It is also called the F-score or F-measure. It is used in deep learning [177]. It conveys the balance between the precision and the recall. It also tells us how many instances it classifies correctly. Its highest possible value is 1, which indicates perfect precision and recall. Its lowest possible value is 0, when either the precision or the recall is zero. It can be formulated as
  (4) $$\begin{array}{c} F1S=\frac{2}{1/PRS+1/RES}=\frac{t_{p}}{t_{p}+f_{p}+f_{n}/2}\text{,} \end{array}$$
where *PRS* is the number of correct positive results divided by the number of positive results predicted with the classifier and *RES* is the number of correct positive results divided by the number of all relevant samples.
(vi) RTM ⇒ Estimating the *RTM* complexity of algorithms is mandatory for many applications (e.g., embedded real-time systems [180]). The optimization of the *RTM* complexity of algorithms in applications is highly expected. The total *RTM* can prove to be one of the most important determinative performance factors in many software-intensive systems.
(vii) GMN ⇒ It indicates the central tendency or typical value of a set of numbers by considering the product of their values instead of using their sum. It can be used to attain a more accurate measure of returns than the mean or arithmetic mean or average. The GMN for any set of numbers *x*_1_, *x*_2_, *x*_3_,…, *x*_*m*_ can be defined as
  (5) $$\begin{array}{c} GMN={\left(\overset{m}{\underset{i=1}{\prod }}x_{i}\right)}^{1/m}=\sqrt{\left[m\right]}x_{1}x_{2}x_{3}\cdots x_{m}\text{.} \end{array}$$
(viii) MCC ⇒ The Matthews correlation coefficient (MCC) is used as a measure of the quality of binary classifications, introduced by biochemist Brian W. Matthews in 1975.
(ix) *κ*⇒ The metric of Cohen's kappa (*κ*) can be used to evaluate binary classifications.

## 3. A Succinct Survey of State of the Art

This section deals with a summary of existing studies apposite for the classification of breast cancer histopathological images followed by a short discussion and our findings.

### 3.1. Summary of Previous Studies

Table 2 provides a short summary of previous studies carried out to classify breast cancer from images. Experimental results of miscellaneous deep models in the literature on publicly available datasets demonstrated various degrees of accurate cancer prediction scores. However, as AUC and ACC are the most important metrics for breast cancer histopathological images classification [49], the experimental results in Table 2 take them into account as the performance indices.

### 3.2. Key Techniques and Challenges

The CNNs can be regarded as a variant of the standard neural networks. Instead of using fully connected hidden layers, the CNNs introduce the structure of a special network, which comprises so-called alternating convolution and pooling layers. They were first introduced for overcoming known problems of fully connected deep neural networks when handling high dimensionality structured inputs, such as images or speech. From Table 2, it is noticeable that CNNs have become state-of-the-art solutions for breast cancer histology images classification. However, there are still challenges even when using the CNN-based approaches to classify pathological breast cancer images [16], as given below:

- Risk of overfitting ⇒ The number of parameters of CNN increases rapidly depending on how large the network is, which may lead to poor learning.
- Being cost-intensive ⇒ To get a huge number of labeled breast cancer images is very expensive.
- Huge training data ⇒ CNNs need to be trained using a lot of images, which might not be easy to find considering that collecting real-world data is a tedious and expensive process.
- Performance degradation ⇒ Various hyperparameters have a significant influence on the performance of the CNN model. The model's parameters need to be tuned properly to achieve a desirable result [75], which usually is not an easy task.
- Employment difficulty ⇒ In the process of training CNN model, it is usually inevitable to rearrange the learning rate parameters to get a better performance. This makes it arduous for the algorithm to use in real-life applications by nonexpert users [181].

Many methods had been proposed in the literature considering the aforementioned challenges. In 2012, AlexNet [81] architecture was introduced for ImageNet Challenge having error rate of 16%. Later various variations of AlexNet [81] with denser network were introduced. Both AlexNet [81] and VGGNet [98] were the pioneering works that demonstrated the potential of deep neural networks [182]. AlexNet was designed by Alex Krizhevsky [81]. It contained 8 layers; the first 5 were convolutional layers, some of them followed by max-pooling layers, and the last 3 were fully connected layers [81]. It was the first large-scale CNN architecture that did well on ImageNet [183] classification. AlexNet [81] was the winner of the ILSVRC [183] classification, the benchmark in 2012. Nevertheless, it was not very deep. SqueezeNet [184] was proposed to create a smaller neural network with fewer parameters that could be easily fit into computer memory and transmitted over a computer network. It achieved AlexNet [81] level accuracy on ImageNet with 50x fewer parameters. It was compressed to less than 0.5 MB (510x smaller than AlexNet [81]) with model compression techniques. The VGG [98] is a deep CNN used to classify images. The VGG19 is a variant of VGG which consists of 19 layers (i.e., 16 convolution layers and 3 fully connected layers, in addition to 5 max-pooling layers and 1 SoftMax layer) [98]. There exist many variants of VGG [98] (e.g., VGG11, VGG16, VGG19, etc.). VGG19 has 19.6 billion FLOPs (floating point operations per second). VGG [98] is easy to implement but slow to train. Nowadays, many deep-learning-based methods are implemented on influential backbone networks; among them, both DenseNet [67] and ResNet [75] are very popular. Due to the longer path between the input layer and the output layer, the information vanishes before reaching its destination. DenseNet [67] was developed to minimize this effect. The key base element of ResNet [75] is the residual block. DenseNet [67] concentrates on making the deep learning networks move even deeper as well as simultaneously making them well organized to train by applying shorter connections among layers. In short, ResNet [75] adopts summation, whereas DenseNet [67] deals with concatenation. Yet, the dense concatenation of DenseNet [67] creates a challenge of demanding high GPU (Graphics Processing Unit) memory and more training time [182]. On the other hand, the identity shortcut that balances training in ResNet [75] curbs its representation dimensions [182]. Compendiously, there is a dilemma in the alternative between ResNet [75] and DenseNet [67] for many applications in terms of performance and GPU resources [182].

### 3.3. Our Findings

Although various deep learning models in Table 2 often achieved pretty good scores of AUC and ACC, the models demand a large amount of data but breast cancer diagnosis always suffers from a lack of data. To adopt artificial data is a tentative solution of this issue, but the determination of the best hyperparameters is extremely difficult. Besides efficient deep learning models, the datasets themselves have some limitations, for example, overinterpretation, which cannot be diagnosed using typical evaluation methods based on the ACC of the model. Deep learning models trained on popular datasets (e.g., BreaKHis [33]) may suffer from overinterpretation. In overinterpretation, deep learning models make confident predictions based on details that do not make any sense to humans (e.g., promiscuous patterns and image borders). When deep learning models are trained on datasets, they can make apparently authentic predictions based on both meaningful and meaningless subtle signals. This effect, eventually, can reduce the overall classification performance of deep models. Most probably, this is one of the reasons why any state-of-the-art deep learning model in the literature for classifying breast cancer histopathological images (see Table 2) could not show an ACC of 100%.

In addition, the training-testing ratio can regulate the performance of a deep model for image classification. We wish to determine the most popular and/or optimized training-testing ratios for classifying histopathological images using Table 2. To this end, we have calculated the usage frequency of the training-testing ratio (i.e., percentage of the number of papers that used the same ratio) by considering data in Table 2 and the following equation:

(6) $$\begin{array}{c} Usagefrequency\left(\%\right)=\frac{\left(Totalnumberofpapersuse\;da\;training-testingratio\right)\left(100\right)}{Sumofpapersbothuse\;da\;ndu\;nuse\;dt\;hesametraining-testingratio}\text{.} \end{array}$$

Figure 3 demonstrates the frequency of usage of training-testing ratio considering data in Table 2. From Figure 3, it is noticeable that the most popular training-testing ratio for histopathological image classification is 70%: 30%. The second-best used training-testing ratio is 80%: 20%, followed by 90%: 10%, 75%: 25%, 50%: 50%, and so on.  Figure 4 presents the GMN of ACC for the most frequently used training-testing ratios considering data in Table 2. It shows a different history; in terms of ACC, the rate of 80%: 20% became the best option for the training-testing ratio to classify histopathological images. Explicitly, the GMN of ACC formed like a Gaussian shaped curve and the ratio of 80%: 20% owned its highest peak. To cut a long story short, by considering ACC, the training-testing ratio of 80%: 20% became the finest and the optimal choice for classifying histopathological images.

## 4. Methods and Materials

This section explains in detail our proposed DenTnet model and its implementation.  Figure 5 demonstrates a general flowchart of our methodology to classify breast cancer histopathological images automatically.

### 4.1. Architecture of Our Proposed DenTnet

The architecture of our proposed DenTnet is shown in Figure 1, which consists of four different blocks, namely, the input volume, training from scratch, transfer learning, and fusion and recognition.

#### 4.1.1. Input Volume

The input is a 3D RGB (three-dimensional red, green, and blue) image with a size of 224 × 224, that is, 224 × 224 × 3.

#### 4.1.2. Training from Scratch

Initially, features are extracted from the input images by feeding the input to the convolutional layer. The convolution (conv) layers contain a set of filters (or kernels) parameters, which are learned throughout the training. The size of the filters is usually smaller than the actual image, where each filter convolves with the image and creates an activation map. Thereafter, the pooling layer progressively decreases the spatial size of the representation for reducing the number of parameters in the network. Instead of differentiable functions such as sigmoid and tanh, the network utilizes the ReLU as an activation function. Finally, the extracted features or the output of the last layer from the training from scratch block is then amalgamated with the features extracted from the transfer learning approach. Figure 1 includes the design of the DenseNet [67] architecture used to extract the feature using the learning-from-scratch approach.

#### 4.1.3. Transfer Learning

In transfer learning, given that a domain *𝒟* consists of feature space *𝒳* and a marginal probability distribution *P*(*X*), where *X* = *x*_1_, *x*_2_,…, *x*_*n*_∈*X*, and a task *𝒯* consists of a label space *𝒴* and an objective predictive function *f*: *𝒳*⟶*𝒴*, the corresponding label *f*(*x*) of a new instance *x* is predicted by function *f*, where the new tasks denoted by *𝒯* = *𝒴*, *f*(*x*) are learned from the training data consisting of pairs *x*_*i*_ and *y*_*i*_, where *x*_*i*_ ∈ *X* and *y*_*i*_ ∈ *𝒴*. When utilizing the learning-from-scratch approach, the extracted features stay in the same distribution. To solve this problem, we amalgamated both learning-from-scratch and the transfer learning approach. The learned parameters are further fine-tuned by retraining the extracted features. This is anticipated to expand the prior knowledge of the network about the data, which might improve the efficiency of the model during training, thereby accelerating the learning speed and also increasing the accuracy of the model. As shown in Figure 1, there is a connection between the blocks of the input volume and transfer learning. The transfer learning approach extracted features from the ImageNet [168] weights. The weight is the parameters (including trainable and nontrainable) learned from the ImageNet [168] dataset. Since transfer learning involves transferring knowledge from one domain to another, we have utilized the ImageNet weight as the models developed in the ImageNet [168] classification competition are measured against each other for performance. Henceforth, the ImageNet weight provides a measure of how good a model is for classification. Besides, the ImageNet weight has already showed a markedly high accuracy [185]. The extracted features are then used by the network before being passed to the fusion and recognition block, where the features are amalgamated with the extracted features from the learning-from-scratch block for recognition.

#### 4.1.4. Fusion and Recognition

The extracted features based on the ImageNet weights are then amalgamated with the features extracted by the block of training from scratch. A global average pooling is performed. Dropout technique helps to prevent a model from overfitting. It is used with dense fully connected layers. The fully connected layer compiles the data extracted by previous layers to form the final output. The last step passes the features through the fully connected layer, which then uses SoftMax to classify the class of the input images.

### 4.2. Implementation Details

#### 4.2.1. Data Preparation

We have adopted data augmentation, stain normalization, and image normalization strategies to optimize the training process. Hereby, we have explained each of them briefly.

#### 4.2.2. Data Augmentation

Due to the limited size of the input samples, the training of our DenTnet was prone to overfitting, which caused low detection rate. One solution to alleviate this issue was the data augmentation, which generated more training data from the existing training set. Dissimilar data augmentation techniques (e.g., horizontal flipping, rotating, and zooming) were applied to datasets for creating more training samples.

#### 4.2.3. Stain Normalization

The breast cancer tissue slices are stained by H&E to differentiate between nuclei stained with purple color and other tissue structures stained with pink and red color to help pathologists analyze the shape of nuclei, density, variability, and overall tissue structure [186]. The H&E staining variability between acquired images exists due to the different staining protocols, scanners, and raw materials. This is a common problem with histological image analysis. Therefore, stain normalization of H&E-stained histology slides was a key step for reducing the color variation and obtaining a better color consistency prior to feeding input images into the DenTnet architecture. Different techniques are available for stain normalization in histological images. We have considered Macenko technique [187] due to its promising performance in many studies to standardize the color intensity of the tissue. This technique was based on a singular value decomposition. A logarithmic function was used to adaptively transform color concentration of the original histopathological image into its optical density (OD) image as *OD*=−log (*I*/*I*_0_), where *OD* hints the matrix of optical density values, *I* belongs to the image intensity in red-green-blue space, and *I*_0_ addresses the illuminating intensity incident on the histological sample.

#### 4.2.4. Intensity Normalization

Intensity normalization was another important preprocessing step. Its primary aim was to get the same range of values for each input image before feeding to the DenTnet. It also speeded up the convergence of DenTnet. Input images were normalized to the standard normal distribution by min-max normalization (i.e., using one of the most popular ways to normalize data) to the intensity range of [0, 1], which can be computed as

(7) $$\begin{array}{c} x_{normalized}=\frac{x-x_{\min}}{x_{\max}-x_{\min}}\text{,} \end{array}$$

where *x*, *x*_min_, and *x*_max_ indicate pixel, minimum, and maximum intensity values of the input image, respectively.

#### 4.2.5. Hardware and Software Requirements

DenTnet was implemented using the TensorFlow and Keras framework [188, 189] and coded in Python using Jupyter Notebook on a Kaggle Private Kernel. The experiment was performed on a machine with the following configuration: Intel® Xeon® CPU @ 2.30 GHz with 16 CPU Cores, 16 GB RAM, and NVIDIA Tesla P100 GPU. We implemented and trained everything on the cloud using Kaggle GPU hours.

#### 4.2.6. Training and Testing Setup

The dataset was divided in a 80%: 20% ratio, where 80% was used for training and the remaining 20% was used for testing. The data used for testing were kept isolated from the training set and never seen by the model during training. To evaluate the images classification, we have computed the recognition rate at the image level over the two different classes: (i) correctly classified images and (ii) the total number of images in the test set.

#### 4.2.7. Training Procedure

In the training of a neural network, a measure of error is required to compute the error between the targeted output and the computed output of training data known as the loss function. An optimization algorithm is needed to minimize this function. We have considered Adam optimizer [190] with numerical stability constant *epsilon* *=* *None, decay* *=* *0.0,* and *AMSGrad* *=* *True*.  Table 3 presents the hyperparameter values of the proposed deep learning model. Learning rate (also referred to as step size) signifies the proportion to which weights are updated. A smaller value (e.g., 0.000001) slows down the learning process during training, whereas a larger value (e.g., 0.400) results in faster learning. We have considered a learning rate of 0.001. The exponential decay rates of the first and second moments were estimated to be 0.60 and 0.90, respectively. To update the weights, the number of epochs was set to 50 with 3222 steps per epoch and a batch size of 32. For the BreaKHis [33] dataset, we had a training sample of 103104 images, with 12288 validation samples and 697 testing samples. The training process used 10-fold cross-validation, where one of the samples was used to validate the data and the remaining 9 samples were used to train the DenTnet model. The fully connected layer used 1024 filters with a dropout rate of 0.50. Finally, the last layer used two filters with a SoftMax layer to classify the image into two classes (e.g., benign and malignant). We have used categorical cross-entropy as the objective function to quantify the difference between two probability distributions. The whole training process took more than 4 hours for the breast cancer tissue images.

## 5. Experimental Results and Comparison on BreaKHis Dataset

This section demonstrates the experimental results achieved from classifying the breast cancer histopathology (i.e., BreaKHis [33]) images using our proposed DenTnet model.

Figure 6 shows the performance curves obtained during the training of DenTnet using BreaKHis [33] dataset. A normalized confusion matrix for the classification of breast cancer test set images is illustrated in Figure 7(a). The main reason for confusion between benign and malignant breast tissues is their similar textures or expression. Henceforth, careful description of texture is required to remove the confusion between the two classes. For binary classification, 5 images only were misclassified, indicating that DenTnet achieved the highest and best ACC of 99.28%. Figures 7(b) and 7(c) demonstrate the ROC curve and precision-recall curve for classification of benign and malignant images from BreaKHis [33] dataset, respectively. AUC of 0.99, sensitivity of 97.73%, and specificity 100% have been reported.  Table 4 lists the complete classification report of DenTnet. It achieved an ACC of 99.28%.

Table 1 compares the results obtained by several methods. The methods of Togacar et al. [26], Parvin et al. [31], Man et al. [36], Soumik et al. [60], Liu et al. [172], Zerouaoui and Idri [56], and Chattopadhyay et al. [174] were centered on mainly CNN models, but they were tested against the same training-testing ratio of 80%: 20% on the BreaKHis dataset [33]. However, Boumaraf et al. [63] suggested a transfer-learning-based method deeming the residual CNN ResNet-18 as a backbone model with block-wise fine-tuning strategy and obtained a mean ACC of 92.15% applying a training-testing ratio of 80%: 20% on BreaKHis dataset [33]. From Table 1, it is notable that DenTnet [ours] achieved the best ACC on the same ground.

## 6. Generalization Ability Evaluation of Proposed DenTnet

What would be the performance of the proposed DenTnet compared with other types of cancer or disease datasets? To evaluate the generalization ability of DenTnet, this section presents the experimental result obtained not only from the dataset of BreaKHis [33] but also from additional datasets of Malaria [191], CovidXray [192], and SkinCancer [193].

### 6.1. Datasets Irrelevant to Breast Cancer

The three following datasets are not related to breast cancer. Herewith, their primary aim is to evaluate the generalization ability of our proposed method DenTnet:

- Malaria [191] ⇒ This dataset contains a total of 27558 infected and uninfected images for malaria.
- SkinCancer [193] ⇒ This dataset contains balanced images from benign skin moles and malignant skin moles. The data consist of two folders, each containing 1800 pictures (224 × 244) from the two types of mole.
- CovidXray [192] ⇒ Corona (COVID-19) virus affects the respiratory system of healthy individual. The chest X-ray is one of the key imaging methods to identify the coronavirus. This dataset contains chest X-ray of healthy versus pneumonia (Corona) infected patients along with few other categories including SARS (Severe Acute Respiratory Syndrome), *Streptococcus*, and ARDS (Acute Respiratory Distress Syndrome) with a goal of predicting and understanding the infection.

Figure 8 specifies some sample images from Malaria [191], SkinCancer [193], and CovidXray [192] datasets.

### 6.2. Experimental Results Comparison

Using four datasets in the experiment, DenTnet has been compared with six widely used and well-known deep learning models, namely, AlexNet [81], ResNet [75], VGG16 [98], VGG19 [98], Inception V3 [88], and SqueezeNet [184]. To evaluate and analyze the performance of DenTnet, four different cases are considered. The first case is the evaluation of different deep learning methods, which are trained and tested on BreaKHis [33] dataset. The second case studies the performance of the deep-learning-based classification methods that are trained and tested on Malaria [191] dataset. The third case is to train and test the deep learning models on SkinCancer [193] dataset. The final one is to understand and analyze the performance of the deep learning models on CovidXray [192] dataset. The overall results are tabulated in Tables 5–9. Besides, the RTM in seconds of various datasets using the deep learning models is shown in Table 10.

According to the results in terms of GMN of ACC, RES, F1S, and AUC as shown in Tables 5–9, respectively, the proposed DenTnet architecture provides the best scores as compared to AlexNet [81], ResNet [75], VGG16 [98], VGG19 [98], Inception V3 [88], and SqueezeNet [184]. On the other hand, DenTnet gets the third best result. Moreover, in most of the cases, AlexNet [81] obtains the lowest results.

### 6.3. Performance Evaluation

The deepening of deep models makes their parameters rise rapidly, which may lead to overfitting of the model. To take the edge off the overfitting problem, predominantly a large number of dataset images are required as the training set. Considering a small dataset, it is possible to reduce the risk of overfitting of the model by reducing the parameters and augmenting the dataset. Accordingly, DenTnet used fewer parameters along with the dense connections in the construction of the model, instead of the direct connections among the hidden layers of the network. As DenTnet used fewer parameters, it attenuated the vanishing gradient descent and strengthened the feature propagation. Consequently, the proposed DenTnet outperformed its alternative state-of-the-art methods. Yet, its runtime was a bit longer in Malaria [191] and SkinCancer [193] datasets as compared to ResNet [75]. The main reason why the DenTnet model may require more time is that it uses many small convolutions in the network, which can run slower on GPU than compact large convolutions with the same number of GFLOPS. Still, DenTnet includes fewer parameters compatibility when compared to ResNet [75]. Henceforth, it is more efficient in solving the problem of overfitting. In general, all of the used algorithms suffered from some degree of overfitting problem on all datasets. We minimized such problems by reducing the batch size and adjusting the learning rate and the dropout rate. In some cases, the proposed DenTnet predicted fewer positive samples as compared to ResNet [75]. This is due to the lack of its conservative designation of the positive class. Thus, the GMN PRS of the proposed DenTnet was about 2% lower than that of ResNet [75].

As VGG16 [98] is easier to implement, many deep learning image classification problems benefit from the technique by using the network either as a sole model or as a backbone architecture to classify images. While VGG19 [98] is better than the VGG16 [98] model, they are both very slow to train—for example, a ResNet with 34 layers only requires 18% of operations as a VGG with 19 layers (around half the layers of the ResNet) will require [194]. Regarding AlexNet [81], the model struggled to scan all features as it is not very deep, resulting in poor performance. The SqueezeNet [184] model achieved approximately the same performance as the AlexNet [81] model. VGG19 [98] and Inception V3 [88] showed almost the same level of effectiveness. Although the ResNet [75] model has proven to be a powerful tool for image classification and is usually fast, it has been shown to take a long time to train. Concisely, using all benefits of DenseNet [67] with optimization, DenTnet obtained the highest GMN ACC of 0.9463, RES of 0.9649, F1S of 0.9531, and AUC of 0.9465 from all four datasets. This implies that DenTnet has the best generalization ability compared to its alternative methods.

Often, it is important to measure that certain deep learning models are more efficient and practical as compared to their alternatives. Seemingly, it is difficult to measure such superiority from the obtained experimental results in Tables 5–10. Nonetheless, nonparametric statistical test can make a clear picture of this issue.

## 7. Nonparametric Statistical Analysis

Figure 9 depicts performance evaluation of various algorithms deeming the numerical values of the ineffectualness metrics and RTM from Table 11. It is noted that, for a better visualization purpose, the RTM scores in Figure 9 use log-normal distribution [195] with a mean of 10 and standard deviation of 1. However, from this graph, it is extremely hard to rank each algorithm. However, statistically, it is possible to show that one algorithm is better than its alternatives. Friedman test [196] and its derivatives (e.g., Iman-Davenport test [197]) are normally referred to as examples of the most well-known nonparametric tests for multiple comparisons. The mathematical equations of Friedman [196], Friedman's aligned rank [198], and Quade [199] tests can be found in the works of Quade [199] and Westfall and Young [200]. Friedman test [196] takes measures in preparation for ranking of a set of algorithms with performance in descending order. But it can solely inform us about the appearance of differences among all samples of results under comparison. Henceforth, its alternatives (e.g., Friedman's aligned rank test [198] and Quade test [199]) can give us further information. Consequently, we have performed the tests of Friedman [196], Friedman's aligned rank [198], and Quade [199] for average rankings based on the features of our experimental study. On rejecting null-hypotheses, we have continued to use post hoc procedures to find the special pairs of algorithms that give idiosyncrasies. In the case of 1 × *N* comparisons, the post hoc procedures make up for Bonferroni-Dunn's [201], Holm's [202], Hochberg's [203], Hommel's [204, 205], Holland and Copenhaver's [206], Rom's [207], Finner's [208], and David Li's [209] procedures, whereas the post hoc procedures of Nemenyi [210], Shaffer [211], and Bergmann-Hommel [212] are involved in *N* × *N* comparisons. The details can be found in the works of Bergmann and Hommel [212], García and Herrera [213], and Hommel and Bernhard [205].

### 7.1. Average Ranking of Algorithms

To get the nonparametric statistical test results, Friedman [196], Friedman's aligned rank [198], and Quade [199] tests have been applied to the results of seven models in Table 11. Explicitly, statistical tests have been applied to a matrix with dimension of 7 × 6, where 7 is the number of models and 6 is the number of parameters (as 6 datasets while applied to the statistical software environment [214]) in each model.  Table 12 shows the average ranking computed by using Friedman [196], Friedman's aligned rank [198], and Quade [199] nonparametric statistical tests. The nonparametric Friedman [196], Friedman's aligned rank [198], and Quade [199] tests determine whether there were significant differences among various models taking data from Table 11. These tests provide the average ranking of all algorithms; that is, the best performing algorithm gets the highest rank of 1, the second-best algorithm gets the rank of 2, and so on.

Figure 10 makes a visualization of the average rankings using the data in Table 12. From Figure 10, it is noticeable that the algorithm of DenTnet [ours] became the best performing one, with the longest bars of 0.6667, 0.1395, and 0.7242 for Friedman test [196], Friedman's aligned rank test [198], and Quade test [199], respectively. This indicates that the algorithm of DenTnet [ours] gives great performance for the solution of underlaying problems of classifying breast cancer histopathological images from four different datasets. Friedman [196] statistic considered reduction performance (distributed according to chi-square with 6 degrees of freedom) of 24.500000. Friedman's aligned [198] statistic considered reduction performance (distributed according to chi-square with 6 degrees of freedom) of 23.102557. Iman-Davenport [197] statistic considered reduction performance (distributed according to F-distribution with 6 and 30 degrees of freedom) of 10.652174. Quade [199] statistic considered reduction performance (distributed according to F-distribution with 6 and 30 degrees of freedom) of 5.274194. The *p* values computed through Friedman statistic, Friedman's aligned statistic, Iman-Davenport statistic, and Quade statistic are 0.000422, 0.000762847204, 0.000002458229, and 0.000820133186, respectively.

Table 13 demonstrates the results obtained on post hoc comparisons of adjusted *p* values; *α*=0.05 and *α*=0.10. Using level of significance *α*=0.05, (i) Bonferroni-Dunn's [201] procedure rejects those hypotheses that have an unadjusted *p* value ≤0.008333; (ii) Holm's [202] procedure rejects those hypotheses that have an unadjusted *p* value ≤0.016667; (iii) Hochberg's [203] procedure rejects those hypotheses that have an unadjusted *p* value ≤0.0125; (iv) Hommel's [204] procedure rejects those hypotheses that have an unadjusted *p* value ≤0.016667; (v) Holland's [206] procedure rejects those hypotheses that have an unadjusted *p* value ≤0.016952; (vi) Rom's [207] procedure rejects those hypotheses that have an unadjusted *p* value ≤0.013109; (vii) Finner's [208] procedure rejects those hypotheses that have an unadjusted *p* value ≤0.033617; and (viii) Li's [209] procedure rejects those hypotheses that have an unadjusted *p* value ≤0.021422.

### 7.2. Post Hoc Procedures: 1 × *N* Comparisons

In the case of 1 × *N* comparisons, the post hoc procedures consist of Bonferroni-Dunn's [201], Holm's [202], Hochberg's [203], Hommel's [204, 205], Holland and Copenhaver's [206], Rom's [207], Finner's [208], and David Li's [209] procedures. In these tests, multiple comparison post hoc procedures have been considered for comparing the control algorithm of DenTnet [ours] with others. The results have been shown by computing *p* values for each comparison.  Table 14 depicts the obtained *p* values using the ranks computed by nonparametric Friedman [196], Friedman's aligned rank [198], and Quade [199] tests. All tests have demonstrated significant improvements of DenTnet [ours] over AlexNet [81], ResNet [75], VGG16 [98], VGG19 [98], Inception V3 [88], and SqueezeNet [184] counting each and every post hoc procedure. Besides, David Li's [209] procedure had the greatest performance, reaching the lowest *p* value in the comparisons.

### 7.3. Post Hoc Procedures: *N* × *N* Comparisons

In the case of *N* × *N* comparisons, the post hoc procedures consist of Nemenyi's [210], Shaffer's [211], and Bergmann-Hommel's [212] procedures.  Table 15 presents 21 hypotheses of equality among 7 different algorithms and *p* values achieved. Using level of significance *α*=0.05, (i) Nemenyi's [210] procedure rejects those hypotheses that have an unadjusted *p* value ≤0.002381; (ii) Holm's [202] procedure rejects those hypotheses that have an unadjusted *p* value ≤0.002778; (iii) Shaffer's [211] procedure rejects those hypotheses that have an unadjusted *p* value ≤0.002381; and (iv) Bergmann's [212] procedure rejects those hypotheses of AlexNet [81] versus DenTnet [ours], ResNet [75] versus SqueezeNet [184], and SqueezeNet [184] versus DenTnet [ours]. On the other hand, considering *α*=0.10, (i) Nemenyi's [210] procedure rejects those hypotheses that have an unadjusted *p* value ≤0.004762; (ii) Holm's [202] procedure rejects those hypotheses that have an unadjusted *p* value ≤0.005556; (iii) Shaffer's [211] procedure rejects those hypotheses that have an unadjusted *p* value ≤0.004762; and (iv) Bergmann's [212] procedure rejects those hypotheses of AlexNet [81] versus DenTnet [ours], ResNet [75] versus SqueezeNet [184], and SqueezeNet [184] versus DenTnet [ours].

### 7.4. Critical Distance Diagram from Nemenyi [210] Test

Nemenyi [210] test is very conservative with a low power, and hence it is not a recommended choice in practice [215]. Nevertheless, it has a unique advantage of having an associated plot to demonstrate the results of fair comparison.  Figure 11 depicts the Nemenyi [210] post hoc critical distance diagrams at three distinct levels of significance *α* values. If the distance between algorithms is less than the critical distance, then there is no statistically significant difference between them. The diagrams in Figures 11(a) and 11(b) associated with *α*=0.10 with the critical distance of 3.3588 and with *α*=0.05 with the critical distance of 3.6768, respectively, are identical, whereas the diagram in Figure 11(c) related to *α*=0.01 with the critical distance of 4.3054 is different. Any two algorithms are considered as significantly different if their performance variation is greater than the critical distance. To this end, from Figure 11, it is noticeable that, at *α*=0.01, both SqueezeNet [184] versus DenTnet [ours] and SqueezeNet [184] versus ResNet [75] are remarkably different, while other pairs are not remarkably divergent as their performance differences are less than 4.3054. As compared to ResNet [75], DenTnet [ours] differs from SqueezeNet [184] by a greater distance. On the other hand, SqueezeNet [184] versus DenTnet [ours] and AlexNet [81] versus DenTnet [ours] are significantly different at both *α*=0.10 and *α*=0.05, whereas SqueezeNet [184] versus ResNet [75] is significantly dissimilar at those *α* values. Straightforwardly, DenTnet [ours] is outstandingly unalike both SqueezeNet [184] and AlexNet [81], but ResNet [75] is not outstandingly unalike AlexNet [81]. This implies that the method of DenTnet [ours] outperforms that of ResNet [75], which also agrees with the finding in Figure 10.

### 7.5. Reasons of Superiority

In this study, DenseNet [67] was a great choice as it was very compact and deep. It used less training parameters and reduced the risk of model overfitting and improved the learning rate. In the dense block of DenTnet, the outputs from the previous layers were concatenated instead of using the summation. This type of concatenation helped to markedly speed up the processing of data for large number of columns. The dense block of DenTnet contained convolution and nonlinear layers, which applied several optimization techniques (e.g., dropout and BN). DenTnet scaled to hundreds of layers, while exhibiting no optimization difficulties. Overall, this model was applied to a very large number of preprocessed augmented images from BreaKHis [33], Malaria [191], SkinCancer [193], and CovidXray [192] datasets. To the best of our knowledge, no other studies in the literature had such an edge. Additionally, the use of data augmentation approach in this study positively affected the performance of the model due to expansion in the size of training data, which is the foremost requirement of a deep network for its proper working. Our DenTnet was well trained through various parameters' tuning. For example, in the case of BreaKHis [33], unlike other existing models, our model was trained on all the magnifications combined (40x, 100x, 200x, and 400x) to avoid any loss of generality.

In sum and substance, based on the aforementioned experimental and nonparametric statistical test results, it is, therefore, possible to conclude that the proposed DenTnet [ours] outperformed AlexNet [81], ResNet [75], VGG16 [98], VGG19 [98], Inception V3 [88], and SqueezeNet [184] in terms of computational speed. Significantly, the accuracy achieved by the proposed DenTnet [ours] surpassed those of existing state-of-the-art models in classifying images of the BreaKHis [33], Malaria [191], SkinCancer [193], and the CovidXray [192] dataset.

### 7.6. Limitation of Proposed Model and Methodology

Despite these promising results, questions remain as to whether the proposed DenTnet model could be utilized to classify categorical images. Moreover, DenTnet was tested with one breast cancer dataset (i.e., BreaKHis [33]) only. Although the generalization ability of DenTnet with three non-breast-cancer-related datasets was studied in Section 6, it is unknown whether DenTnet can generalize to other state-of-the-art breast cancer datasets. Future work should, therefore, investigate the efficacy and generalizability of DenTnet with datasets along with multiclass labels, as well as other publicly available breast cancer datasets (e.g., the most recently introduced MITNET dataset [216]).

The classification effect of breast cancer histopathological images of any deep learning methodology is related to the features and many studies predominantly focused on how to develop good feature descriptors and better extract features. Different from traditional handcrafted feature-based models, DenTnet can automatically extract more abstract features. Nevertheless, it is worth noting that although the proposed DenTnet has addressed the cross-domain problem by utilizing the transfer learning approach, features extracted in the methodology are solely deep-network-based features, which are extracted by feeding images directly to the model. However, feeding deep models directly with images would not generalize as the models consider color distribution of an image. It is understood that local information can be captured from color images using Local Binary Pattern (LBP) [217]. Therefore, future work can use multiple types of features by combining the features extracted by the proposed method with LBP features to address this issue.

## 8. Conclusion

We presented that, for classifying breast cancer histopathological images, the most popular training-testing ratio was 70%: 30%, while the best performance was indicated by the training-testing ratio of 80%: 20%. We proposed a novel approach named DenTnet to classify histopathology images using training-testing ratio of 80%: 20%. DenTnet achieved a very high classification accuracy on the BreaKHis dataset. Several impediments of existing state-of-the-art methods including the requirement of high computation and the utilization of the identical feature distribution were attenuated. To test the generalizability of DenTnet, we conducted experiments on three additional datasets (Malaria, SkinCancer, and CovidXray) with varying difficulties. Experimental results on all four datasets demonstrated that DenTnet achieved a better performance in terms of accuracy and computational speed than a large number of effective state-of-the-art classification methods (AlexNet, ResNet, VGG16, VGG19, InceptionV3, and SqueezeNet). These findings contributed to our understanding of how a lightweight model could be used to improve the accuracy and accelerate the learning process of images, including histopathology image classification on using the wild state-of-the-art datasets. Future work shall investigate the efficacy of DenTnet on datasets with multiclass labels.

## Figures and Tables

**Figure 1:** Architecture of the proposed DenTnet.

**Figure 2:** A sample breast cancer histopathological image [79] with four magnification levels of (a) 40x, (b) 100x, (c) 200x, and (d) 400x.

**Figure 3:** Determination of the most popular training-testing ratios using data from Table 2.

**Figure 4:** GMN of ACC for the most popular training-testing ratios deeming data from Table 2.

**Figure 5:** Flowchart of our methodology to classify breast cancer histopathological images.

**Figure 6:** (a) hints ACC and (b) shows loss charts of DenTnet during training.

**Figure 7:** (a) hints confusion matrix for benign and malignant classification, (b) shows ROC curve, and (c) demonstrates precision-recall curve.

**Figure 8:** (a), (b), and (c) specify images of Malaria [191], SkinCancer [193], and CovidXray [192] datasets, respectively.

**Figure 9:** Plotting of the numerical values using data from Table 11.

**Figure 10:** Plotting of average rankings data from Table 12, where each value *x* is plotted as 1/*x* to visualize the highest ranking with the tallest bar.

**Figure 11:** Nemenyi [210] post hoc critical distance diagrams for three *α* values using data in Table 11.

**Table 1:** Comparison of results of various methods using training-testing ratio of 80%: 20% on BreaKHis [33]. The best result is shown in bold.

Year	Method	PRS	RES	F1S	AUC	ACC (%)
2020	Togacar et al. [26]	—	—	—	—	97.56
	Parvin et al. [31]	—	—	—	—	91.25
	Man et al. [36]	—	—	—	—	91.44

2021	Boumaraf et al. [63]	—	—	—	—	92.15
	Soumik et al. [60]	—	—	—	—	98.97

2022	Liu et al. [172]	—	—	—	—	96.97
	Zerouaoui and Idri [56]	—	—	—	—	93.85
	Chattopadhyay et al. [174]	—	—	—	—	96.10
	DenTnet [ours]	0.9700	0.9896	0.9948	0.99	**99.28**

**Table 2:** A succinct survey of deep-learning-based histopathological image classification methods. NA indicates either “not available” or “no answer” from the associated authors.

Year	Ref	Aim	Technique	Dataset	Sample	Training (%)	Testing (%)	Result	Performance	
									AUC	ACC
2016	Chan and Tuszynski [80]	To predict tumor malignancy in breast cancer	Employed binarization, fractal dimension, SVM	BreaKHis [33]	7909	50	50	ACC of 97.90%, 16.50%, 16.50%, and 25.30% obtained for 40x, 100x, 200x, and 400x magnification factors, respectively	NA	39.05%
	Spanhol et al. [33]	To classify histopathological images	Employed CNN based on AlexNet [81]	BreaKHis [33]	7909	70	30	ACC of 90.0%, 88.4%, 84.6%, and 86.1% obtained for 40x, 100x, 200x, and 400x magnification factors, respectively	NA	87.28%
	Bayram-oglu et al. [38]	To classify breast cancer histopathology images	Employed single-task CNN and multitask CNN	BreaKHis [33]	7909	70	30	For single-task CNN, ACC of 83.08%, 83.17%, 84.63%, and 82.10%, obtained for 40x, 100x, 200x, and 400x magnification factors, respectively; accordingly, for multitask CNN, ACC of 81.87%, 83.39%, 82.56%, and 80.69%	NA	82.69%
	Abbas [77]	To diagnose breast masses	Applied SURF [82], LBPV [83]	DDSM [84], MIAS [85]	600	40	60	Overall 92%, 84.20%, 91.50%, and 0.91 obtained for sensitivity, specificity, ACC, and AUC, respectively	0.91	91.50%

2017	Song et al. [21]	To classify histopathology images	Employed a model of CNN, Fisher vector [86], SVM	BreaKHis [33], IICBU2008 [87]	8283	70	30	ACC of 94.42%, 89.49%, 87.25%, and 85.62% obtained for 40x, 100x, 200x, and 400x magnification factors, respectively	NA	89.19%
	Wei et al. [22]	To analyze tissue images	Employed a modification of GoogLeNet [88]	BreaKHis [33]	7909	75	25	ACC of 97.46%, 97.43%, 97.73%, and 97.74% obtained for 40x, 100x, 200x, and 400x magnification factors, respectively	NA	97.59%
	Das et al. [23]	To classify histopathology images	Employed GoogLeNet [88]	BreaKHis [33]	7909	80	20	ACC of 94.82%, 94.38%, 94.67%, and 93.49% obtained for 40x, 100x, 200x, and 400x magnification factors, respectively	NA	94.34%
	Kahya et al. [89]	To identify features of breast cancer	Employed dimensionality reduction, adaptive sparse SVM	BreaKHis [33]	7909	70	30	ACC of 94.97%, 93.62%, 94.54%, and 94.42% obtained for 40x, 100x, 200x, and 400x magnification factors, respectively	NA	94.38%
	Song et al. [24]	To classify histopathology images easily	Employed CNN-based Fisher vector [86], SVM	BreaKHis [33]	7909	70	30	ACC of 90.02%, 88.90%, 86.90%, and 86.30% obtained for 40x, 100x, 200x, and 400x magnification factors, respectively	NA	88.03%
	Gupta and Bhavsar [90]	To classify histopathology images.	Employed an integrated model	BreaKHis [33]	7909	70	30	Average ACC of 88.09% and 88.40% obtained for image and patient levels, respectively	NA	88.25%
	Dhungel et al. [91]	To analyze masses in mammograms	Applied multiscale deep belief nets	INbreast [92]	410	60	20	The best results on the testing set with an ACC got 95% on manual and 91% on the minimal user intervention setup	0.76	91.03%
	Spanhol et al. [34]	To classify breast cancer images	Using deep CNN	BreaKHis [33]	7900	70	30	ACC of 84.30%, 84.35%, 85.25% and 82.10% obtained for 40x, 100x, 200x, and 400x magnification factors, respectively	NA	83.96%
	Han et al. [35]	To study breast cancer multiclassification	Employed class structure based CNN	BreaKHis [33]	7909	50	50	ACC of 95.80%, 96.90%, 96.70%, and 94.9% obtained for 40x, 100x, 200x, and 400x magnification factors, respectively	NA	96.08%
	Sun and Binder [39]	To assess performance of H&E stain dat.	A comparative study among ResNet-50 [75], CaffeNet [93], and GoogLeNet [88]	BreaKHis [33]	7909	70	30	ACC of 85.75%, 87.03%, and 84.18% obtained for GoogLeNet [88], ResNet-50 [75], and CaffeNet [93], respectively	NA	85.65%
	Kaymak et al. [94]	To organize breast cancer images	Back-Propagation [95] and Radial Basis Neural Networks [96]	176 images from a hospital	176	65	35	Overall ACC of 59.0% and 70.4% got from Back-Propagation [95] and Radial Basis [96], respectively	NA	64.70%
	Liu et al. [47]	To detect cancer metastases in images	Employed a CNN architecture	Camelyon16 [97]	110	68	32	An AUC of 97.60 (93.60, 100) obtained on par with Camelyon16 [97] test set performance	0.97	95.00%
	Zhi et al. [57]	To diagnose breast cancer images	Employed a variation of VGGNet [98]	BreaKHis [33]	7909	80	20	ACC of 91.28%, 91.45%, 88.57%, and 84.58% obtained for 40x, 100x, 200x, and 400x magnification factors, respectively	NA	88.97%
	Chang et al. [58]	To solve the limited amount of training data	Employed CNN model from Inception [88] family (e.g., Inception V3)	BreaKHis [33]	4017	70	30	ACC of 83.00% for benign class and 89.00% for malignant class. AUC of malignant was 93.00% and AUC of benign was also 93.00%	0.93	86.00%

2018	Jannesari et al. [6]	To classify breast cancer images	Employed variations of Inception [88], ResNet [75]	BreaKHis [33], 6402 images from TMA [99]	14311	85	15	With ResNets ACC of 99.80%, 98.70%, 94.80%, and 96.40% obtained for four cancer types. Inception V2 with fine-tuning all layers got ACC of 94.10%	0.99	96.34%
	Bardou et al. [7]	To classify breast cancer based on histology images	Employed CNN topology, data augmentation	BreaKHis [33]	7909	70	30	ACC of 98.33%, 97.12%, 97.85%, and 96.15% obtained for 40x, 100x, 200x, and 400x magnification factors, respectively	NA	97.36%
	Kumar and Rao [9]	To train CNN for using image classification	Employed CNN topology	BreaKHis [33]	7909	70	30	ACC of 85.52%, 83.60%, 84.84%, and 82.67% obtained for 40x, 100x, 200x, and 400x magnification factors, respectively	NA	84.16%
	Das et al. [11]	To classify breast histopathology images	Employed variation of CNN model	BreaKHis [33]	7909	80	20	ACC of 89.52%, 89.06%, 88.84%, and 87.67% obtained for 40x, 100x, 200x, and 400x magnification factors, respectively	NA	88.77%
	Nahid et al. [100]	To classify biomedical breast cancer images	Employed Boltzmann machine [101], Tamura et al. features [102]	BreaKHis [33]	7909	70	30	ACC of 88.70%, 85.30%, 88.60%, and 88.40% obtained for 40x, 100x, 200x, and 400x magnification factors, respectively	NA	87.75%
	Badejo et al. [103]	To classify medical images	Employed local phase quantization, SVM	BreaKHis [33]	7909	70	30	ACC of 91.10%, 90.70%, 86.20%, and 84.30% obtained for 40x, 100x, 200x, and 400x magnification factors, respectively	NA	88.08%
	Alireza-zadeh et al. [104]	To arrange breast cancer images	Threshold adjacency [105], quadratic analysis [106]	BreaKHis [33]	7909	70	30	ACC of 89.16%, 87.38%, 88.46%, and 86.68% obtained for 40x, 100x, 200x, and 400x magnification factors, respectively	NA	87.92%
	Du et al. [13]	To distribute breast cancer images	Employed AlexNet [81]	BreaKHis [33]	7909	70	30	ACC of 90.69%, 90.46%, 90.64%, and 90.96% obtained for 40x, 100x, 200x, and 400x magnification factors, respectively	NA	90.69%
	Gandom-kar et al. [14]	To model CNN for breast cancer image diagnosis	Employed a variation of ResNet [75] (e.g., ResNet152)	BreaKHis [33]	7786	70	30	ACC of 98.60%, 97.90%, 98.30%, and 97.60% obtained for 40x, 100x, 200x, and 400x magnification factors, respectively	NA	98.10%
	Gupta and Bhavsar [15]	To model CNN for breast cancer image diagnosis	Employed DenseNet [67], XGBoost classifier [107]	BreaKHis [33]	7909	70	30	ACC of 94.71%, 95.92%, 96.76%, and 89.11% obtained for 40x, 100x, 200x, and 400x magnification factors, respectively	NA	94.12%
	Ben-hammou et al. [17]	To study CNN for breast cancer images	Employed Inception V3 [88] module	BreaKHis [33]	7909	70	30	ACC of 87.05%, 82.80%, 85.75%, and 82.70% obtained for 40x, 100x, 200x, and 400x magnification factors, respectively	NA	84.58%
	Morillo et al. [108]	To label breast cancer images	Employed KAZE features [109]	BreaKHis [33]	7909	70	30	ACC of 86.15%, 80.70%, 77.95%, and 72.00% obtained for 40x, 100x, 200x, and 400x magnification factors, respectively	NA	97.20%
	Chattoraj and Vishwakarma [110]	To study breast carcinoma images	Zernike moments [111], entropies of Renyi [112], Yager [113]	BreaKHis [33]	7909	70	30	ACC of 87.7%, 85.8%, 88.0%, and 84.6% obtained for 40x, 100x, 200x, and 400x magnification factors, respectively	NA	96.53%
	Sharma and Mehra [19]	To analyze behavior of magnification independent breast cancer	Employed models of VGGNet [98] and ResNet [75] (e.g., VGG16, VGG19, and ResNet50)	BreaKHis [33]	7909	90	10	Pretrained VGG16 with logistic regression classifier showed the best performance with 92.60% ACC, 95.65% AUC, and 95.95% ACC precision score for 90%–10% training-testing data splitting	0.95	94.28%
	Zheng et al. [114]	To study content-based image retrieval	Employed binarization encoding, Hamming distance [115]	BreaKHis [33] and others	16309	70	30	ACC of 47.00%, 40.00%, 40.00%, and 37.00% obtained for 40x, 100x, 200x, and 400x magnification factors, respectively	NA	41.00%
	Cascianelli et al. [20]	To study features extraction from images	Employed dimensionality reduction using CNN	BreaKHis [33]	7909	75	25	ACC of 84.00%, 88.20%, 87.00%, and 80.30% obtained for 40x, 100x, 200x, and 400x magnification factors, respectively	NA	84.88%
	Mukkamala et al. [116]	To study deep model for feature extraction	Employed PCANet [117]	BreaKHis [33]	7909	80	20	ACC of 96.12%, 97.41%, 90.99%, and 85.85% obtained for 40x, 100x, 200x, and 400x magnification factors, respectively	NA	92.59%
	Mahraban Nejad et al. [51]	To retrieve breast cancer images	Employed a variation of VGGNet [98], SVM	BreaKHis [33]	7909	98	02	An average ACC of 80.00% was demonstrated from BreaKHis [33]	NA	80.00%
	Rakhlin et al. [118]	To analyze breast cancer images	Several deep neural networks and gradient boosted trees classifier	BACH [78]	400	75	25	For 4-class classification task ACC was 87.2% but for 2-class classification ACC was reported to be 93.8%	0.97	90.50%
	Almasni et al. [119]	To detect breast masses	Applied regional deep learning technique	DDSM [84]	600	80	20	Distinguished between benign and malignant lesions with an overall ACC of 97%	0.96	97.00%

2019	Kassani et al. [8]	To use deep learning for binary classification of breast histology images	Usage of VGG19 [98], MobileNet [120], and DenseNet [67]	BreaKHis [33], ICIAR2018 [78], PCam [121], Bioimaging2015 [122]	8594	87	13	Multimodel method got better predictions than single classifiers and other algorithms with ACC of 98.13%, 95.00%, 94.64% and 83.10% obtained for BreaKHis [33], ICIAR2018 [78], PCam [121], and Bioimaging2015 [122], respectively	NA	92.72%
	Alom et al. [10]	To classify breast cancer from histopathological images	Inception recurrent residual CNN	BreaKHis [33], Bioimaging2015 [122]	8158	70	30	From BreaKHis [33], ACC of 97.90%, 97.50%, 97.30%, and 97.40%, obtained for 40x, 100x, 200x, and 400x magnification factors, respectively	0.98	97.53%
	Nahid and Kong [12]	To classify histopathological breast images	Employed RGB histogram [123] with CNN	BreaKHis [33]	7909	85	15	ACC of 95.00%, 96.60%, 93.500%, and 94.20% obtained for 40x, 100x, 200x, and 400x magnification factors, respectively	NA	94.68%
	Jiang et al. [16]	To use CNN for breast cancer histopathological images	Employed CNN, Squeeze-and-Excitation [124] based ResNet [75]	BreaKHis [33]	7909	70	30	The achieved accuracy between 98.87% and 99.34% for the binary classification as well as between 90.66% and 93.81% for the multiclass classification	0.99	95.67%
	Sudharshan et al. [18]	To use instance learning for image sorting	Employed CNN-based multiple instance learning algorithm	BreaKHis [33]	7909	70	30	ACC of 86.59%, 84.98%, 83.47%, and 82.79% obtained for 40x, 100x, 200x, and 400x magnification factors, respectively	NA	84.46%
	Gupta and Bhavsar [25]	To segment breast cancer images	Employed ResNet [75] for multilayer feature extraction	BreaKHis [33]	7909	70	30	ACC of 88.37%, 90.29%, 90.54%, and 86.11% obtained for 40x, 100x, 200x, and 400x magnification factors, respectively	NA	88.82%
	Vo et al. [125]	To extract visual features from training images	Combined weak classifiers into a stronger classifier	BreaKHis [33], Bioimaging2015 [122]	8194	87	13	ACC of 95.10%, 96.30%, 96.90%, and 93.80% obtained for 40x, 100x, 200x, and 400x magnification factors, respectively	NA	95.56%
	Qi et al. [32]	To organize breast cancer images	Employed a CNN network to complete the classification task	BreaKHis [33]	7909	70	30	ACC of 91.48%, 92.20%, 93.01%, and 92.58% obtained for 40x, 100x, 200x, and 400x magnification factors, respectively	NA	92.32%
	Talo [41]	To detect and classify diseases in images	DenseNet [67], ResNet [75] (e.g., DenseNet161, ResNet50)	KimiaPath24 [126]	25241	80	20	DenseNet161 pretrained and ResNet50 achieved ACC of 97.89% and 98.87% on grayscale and color images, respectively	NA	98.38%
	Li et al. [127]	To detect invading component in cancer images	Convolutional autoencoder-based contrast pattern mining framework	361 samples of the breast cancer	361	90	10	ACC was taken into account. The overall ACC achieved was 76.00%, whereas 77.70% was presented for F1S	NA	76.00%
	Ragab et al. [44]	To detect breast cancer from images	AlexNet [81] and SVM	DDSM [84], CBIS-DDSM [128]	2781	70	30	The deep CNN presented an ACC of 73.6%, whereas the SVM demonstrated an ACC of 87.2%	0.88	73.60%
	Romero et al. [45]	To study cancer images	A modification of Inception module [88]	HASHI [129]	151465	63	37	From deep learning networks, an overall ACC of 89.00% was demonstrated along with F1S of 90.00%	0.96	89.00%
	Minh et al. [46]	To diagnose breast cancer images	A modification of ResNet [75] and InceptionV3 [88]	BACH [78]	400	70	20	ACC with 95% for 4 types of cancer classes and ACC with 97.5% for two combined groups of cancer	0.97	96.25%

2020	Stanitsas et al. [130]	To visualize a health system for clinicians	Employed region covariance [131], SVM, multiple instance learning [132]	FABCD [133], BreaKHis [33]	7949	70	15	ACC of 91.27% and 92.00% at the patient and image level, respectively	0.98	91.64%
	Togacar et al. [26]	To analyze breast cancer images rapidly	Employed a ResNet [75] architecture with attention modules	BreaKHis [33]	7909	80	20	ACC of 97.99%, 97.84%, 98.51%, and 95.88% obtained for 40x, 100x, 200x, and 400x magnification factors, respectively	NA	97.56%
	Asare et al. [134]	To study breast cancer images	Employed self-training and self-paced learning	BreaKHis [33]	7909	70	30	ACC of 93.58%, 91.04%, 93.38%, and 91.00% obtained for 40x, 100x, 200x, and 400x magnification factors, respectively	NA	92.25%
	Gour et al. [28]	To diagnose breast cancer tumors images	Employed a modification of ResNet [75]	BreaKHis [33]	7909	70	30	ACC of 90.69%, 91.12%, 95.36%, and 90.24% obtained for 40x, 100x, 200x, and 400x magnification factors, respectively	0.91	92.52%
	Li et al. [29]	To grade pathological images	Employed a modification of Xception network [135]	BreaKHis [33], VLAD [136], LSC [137]	8583	60	40	ACC of 95.13%, 95.21%, 94.09%, and 91.42% obtained for 40x, 100x, 200x, and 400x magnification factors, respectively	NA	93.96%
	Feng et al. [138]	To allocate breast cancer images	Deep neural-network-based manifold preserving autoencoder [139]	BreaKHis [33]	7909	70	30	ACC of 90.12%, 88.89%, 91.57%, and 90.25% obtained for 40x, 100x, 200x, and 400x magnification factors, respectively	NA	90.53%
	Parvin and Mehedi Hasan [31]	To study CNN models for cancer images	LeNet [140], AlexNet [81], VGGNet [98], ResNet [75], Inception V3 [88]	BreaKHis [33]	7909	80	20	ACC of 89.00%, 92.00%, 94.00% and 90.00% obtained for 40x, 100x, 200x, and 400x magnification factors, respectively	0.85	91.25%
	Carvalho et al. [141]	To classify histological breast images	Entropies of Shannon [142], Renyi [112], Tsallis [143]	BreaKHis [33]	4960	70	30	ACC of 95.40%, 94.70%, 97.60%, and 95.50% obtained for 40x, 100x, 200x, and 400x magnification factors, respectively	0.99	95.80%
	Li et al. [144]	To analyze breast cancer images	Employed global covariance pooling module [145]	BreaKHis [33]	7909	70	30	ACC of 96.00%, 96.16%, 98.01%, and 95.97% obtained for 40x, 100x, 200x, and 400x magnification factors, respectively	NA	94.93%
	Man et al. [36]	To classify cancer images	Usage of generative adversarial networks, DenseNet [67]	BreaKHis [33]	7909	80	20	ACC of 97.72%, 96.19%, 86.66%, and 85.18% obtained for 40x, 100x, 200x, and 400x magnification factors, respectively	NA	91.44%
	Kumar et al. [37]	To classify human breast cancer and canine mammary tumors	Employed a framework based on a variant of VGGNet [98] (e.g., VGGNet16) and SVM	BreaKHis [33] and CMTHis [37]	8261	70	30	For BreaKHis [33], ACC of 95.94%, 96.22%, 98.15%, and 94.41% obtained for 40x, 100x, 200x, and 400x magnification factors, respectively; the same for CMTHis [37], ACC of 94.54%, 97.22%, 92.07%, and 82.84% obtained	0.95	96.93%
	Kaushal and Singla [40]	To detect cancerous cells in images.	Employed a CNN model of self-training and self-paced learning	Total 50 images of various patients	50	90	10	ACC was taken into account. Estimation of the standard error of mean was approximately 0.81	NA	93.10%
	Hameed et al. [43]	To use deep learning for classification of breast cancer images	Variants of VGGNet [98] (e.g., fully trained VGG16, fine-tuned VGG16, fully trained VGG19, and fine-tuned VGG19 models)	Breast cancer images: 675 for training and 170 for testing	845	80	20	The ensemble of fine-tuned VGG16 and VGG19 models offered sensitivity of 97.73% for carcinoma class and overall accuracy of 95.29%. It also offered an F1 score of 95.29%	NA	95.29%
	Alantari et al. [48]	To detect breast lesions in digital X-ray mammograms	Adopted three deep CNN models	INbreast [92], DDSM [84]	1010	70	20	In INbreast [92] mean ACC of 89%, 93%, and 95% for CNN, ResNet50, and Inception-ResNet V2, respectively; 95%, 96%, and 98% for DDSM [146]	0.96	94.08%
	Zhang et al. [49]	To classify breast mass	ResNet [75], DenseNet [67], VGGNet [98]	CBIS-DDSM [128], INbreast [92]	3168	70	30	Overall ACC of 90.91% and 87.93% obtained from CBIS-DDSM [128] and INbreast [92], respectively	0.96	89.42%
	Hassan et al. [59]	To classify breast cancer masses	Modification of AlexNet [22] and GoogLeNet [88]	CBIS-DDSM [128], MIAS [85], INbreast [92], etc	600	75	17	With CBIS-DDSM [128] and INbreast [92] databases, the modified GoogLeNet achieved ACC of 98.46% and 92.5%, respectively	0.97	96.98%

2021	Li et al. [147]	To use high-resolution info of images	Multiview attention-guided multiple instance detection network	BreaKHis [33], BACH [78], PUIH [148]	12329	70	30	Overall ACC of 94.87%, 91.32%, and 90.45% obtained from BreaKHis [33], BACH [78], and PUIH [148], respectively	0.99	92.21%
	Wang et al. [27]	To divide breast cancer images	Employed a model of CNN and CapsNet [149]	BreaKHis [33]	7909	70	30	ACC of 92.71%, 94.52%, 94.03%, and 93.54% obtained for 40x, 100x, 200x, and 400x magnification factors, respectively	NA	93.70%
	Albashish et al. [30]	To analyze VGG16 [98]	Employed a variation of VGGNet [98]	BreaKHis [33]	7909	90	10	ACC of 96%, 95.10%, and 87% obtained for polynomial SVM, Radial Basis SVM, and k-nearest neighbors, respectively	NA	92.70%
	Kundale et al. [150]	To classify breast cancer from histology images	Employed SURF [82], DSIFT [151], linear coding [152]	BreaKHis [33]	7909	70	30	ACC of 93.35%, 93.86%, 93.73%, and 94.00% obtained for 40x, 100x, 200x, and 400x magnification factors, respectively	NA	93.74%
	Attallah et al. [153]	To classify breast cancer from histopathological images	Employed several deep learning techniques including autoencoder [139]	BreaKHis [33], ICIAR2018 [78]	7909	70	30	For BreaKHis [33], ACC of 99.03%, 99.53%, 98.08%, and 97.56% got for 40x, 100x, 200x, and 400x magnification factors, respectively; for ICIAR2018 [78], ACC was 97.93%	NA	98.43%
	Burçak et al. [154]	To classify breast cancer histopathological images	Stochastic [155], Nesterov [156], Adaptive [157], RMSprop [158], AdaDelta [159], Adam [160]	BreaKHis [33]	7909	70	30	ACC was taken into account. The overall ACC of 97.00%, 97.00%, 96.00%, and 96.00% obtained for 40x, 100x, 200x, and 400x magnification factors, respectively	NA	96.50%
	Hirra et al. [161]	To label breast cancer images	Patch-based deep belief network [162]	HASHI [129]	584	52	30	Images from four different data samples achieved an accuracy of 86%	NA	86.00%
	Elmannai et al. [42]	To extract eminent breast cancer image features	A combination of two deep CNNs	BACH [78]	400	60	20	The overall ACC for the subimage classification was 97.29% and for the carcinoma cases the sensitivity achieved was 99.58%	NA	97.29%
	Baker and Abu Qutaish [163]	To segment breast cancer images	Clustering and global thresholding methods	BACH [78]	400	70	30	The maximum ACC obtained from classifiers and neural network using BACH [78] to detect breast cancer	NA	63.66%
	Soumik et al. [60]	To classify breast cancer images	Employed Inception V3 [88]	BreaKHis [33]	7909	80	20	ACC of 99.50%, 98.90%, 98.96% and 98.51% obtained for 40x, 100x, 200x, and 400x magnification factors, respectively	NA	98.97%
	Brancati et al. [50]	To analyze gigapixel histopathological images	Employed CNN with a compressing path and a learning path	Camelyon16 [164], TUPAC16 [165]	892	68	32	AUC values of 0.698, 0.639, and 0.654 obtained for max-pooling, average pooling, and combined attention maps, respectively	0.66	NA
	Mahmoud et al. [61]	To classify breast cancer images	Employed transfer learning	Mammography images [166]	7500	80	20	Maximum ACC of 97.80% was claimed by using the given dataset [166]. Sensitivity and specificity were estimated	NA	94.45%
	Munien et al. [62]	To classify breast cancer images	Employed EfficientNet [167]	ICIAR2018 [78]	400	85	15	Overall ACC of 98.33% obtained from ICIAR2018 [78]. Sensitivity was also taken into account	NA	98.33%
	Boumaraf et al. [63]	To analyze breast cancer images	Employed ResNet [75] on ImageNet [168] images	BreaKHis [33]	7909	80	20	ACC of 94.49%, 93.27%, 91.29%, 89.56% obtained for 40x, 100x, 200x, and 400x magnification factors, respectively	NA	92.15%
	Saber et al. [64]	To detect breast cancer	Employed transfer learning technique	MIAS [85]	322	80	20	Overall ACC, PRS, F1S, and AUC of 98.96%, 97.35%, 97.66%, and 0.995, respectively, got from MIAS [85]	0.995	98.96%

2022	Ameh Joseph et al. [169]	To classify breast cancer images	Employed handcrafted features and dense layer	BreaKHis [33]	7909	90	10	ACC of 97.87% for 40x, 97.60% for 100x, 96.10% for 200x, and 96.84% for 400x demonstrated from BreaKHis [33]	NA	97.08%
	Reshma et al. [52]	To detect breast cancer	Employed probabilistic transition rules with CNN	BreaKHis [33]	7909	90	10	ACC, PRS, RES, F1S, and GMN of 89.13%, 86.23%, 81.47%, 85.38%, and 85.17% demonstrated from BreaKHis [33]	NA	89.13%
	Huang et al. [53]	To detect nuclei on breast cancer	Employed mask-region-based CNN	H&E images of patients	537	80	20	PRS, RES, and F1S of 91.28%, 87.68%, and 89.44% demonstrated from the used dataset	NA	95.00%
	Chhipa et al. [170]	To learn efficient representations	Employed magnification prior contrastive similarity	BreaKHis [33]	7909	70	30	Maximum mean ACC of 97.04% and 97.81% were got from patient and image levels, respectively using BreaKHis [33]	NA	97.42%
	Zou et al. [171]	To classify breast cancer images	Employed channel attention module with nondimensionality reduction	BreaKHis [33], BACH [78]	8309	90	10	Average ACC, PRS, RES, and F1S of 97.75%, 95.19%, 97.30%, and 96.30% obtained from BreaKHis [33], respectively. ACC of 85% got from BACH [78]	NA	91.37%
	Liu et al. [172]	To classify breast cancer images	Employed autoencoder and Siamese framework	BreaKHis [33]	7909	80	20	Average ACC, PRS, RES, F1S, and RTM of 96.97%, 96.47%, 99.15%, 97.82%, and 335 seconds obtained from BreaKHis [33], respectively	NA	96.97%
	Jayandhi et al. [54]	To diagnose breast cancer	Employed VGG [98] and SVM	MIAS [85]	322	80	20	Maximum ACC of 98.67% obtained from MIAS [85]. Sensitivity and specificity were also calculated	NA	98.67%
	Sharma and Kumar [55]	To classify breast cancer images	Employed Xception [135] and SVM	BreaKHis [33]	2000	75	25	Average ACC, PRS, RES, F1S, and AUC of 95.58%, 95%, 95%, 95%, and 0.98 obtained from BreaKHis [33], respectively	0.98	95.58%
	Zerouaoui and Idri [56]	To classify breast cancer images	Employed multilayer perceptron, DenseNet201 [67]	BreaKHis [33] and others	NA	80	20	ACC of 92.61%, 92%, 93.93%, and 91.73% on four magnification factors of BreaKHis [33]	NA	93.85%
	Soltane et al. [65]	To classify breast cancer images	Employed ResNet [75]	323 colored lymphoma images	323	50	50	A total of 27 misclassifications for 323 samples were claimed. PRS, RES, F1S, and Kappa score were estimated	NA	91.6%
	Naik et al. [173]	To analyze breast cancer images	Employed random forest, k-nearest neighbors, SVM	699 whole-slide images	699	80	20	Random forest algorithm achieved better result for classifying benign and malignant images from 190 testing samples	NA	98.2%
	Chattopadhyay et al. [174]	To classify breast cancer images	Employed dense residual dual-shuffle attention network	BreaKHis [33]	7909	80	20	Average ACC, PRS, RES, and F1S of 96.10%, 96.03%, 96.08%, and 96.02%, respectively, obtained from four different magnification levels of BreaKHis [33]	NA	96.10%
	Alruwaili and Gouda [66]	To detect breast cancer	Employed the principle of transfer learning, ResNet [75]	MIAS [85]	322	80	20	Best results for ACC, PRS, RES, F1S, and AUC of 89.5%, 89.5%, 90%, and 89.5% obtained from MIAS [85], respectively	NA	89.5%

**Table 3:** List of hyperparameter values for the proposed deep learning model.

Model	Hyperparameters							
	Beta_1	Beta_2	Learning rate	Epoch	Batch size	Epsilon	Decay	AMSGrad
DenTnet	0.60	0.90	0.001	50	32	None	0.0	True

**Table 4:** Classification results by counting all evaluation criteria.

Type	PRS	RES	F1S	Support
Benign	0.98	1.00	0.99	216
Malignant	1.00	0.99	0.99	481
Micro mean	0.99	0.99	0.99	697
Macro mean	0.99	0.99	0.99	697
Weighted mean	0.99	0.99	0.99	697

**Table 5:** ACC of various methods deeming four different datasets.

Models	ACC of various datasets				GMN of ACC	
	BreaKHis [33]	Malaria [191]	SkinCancer [193]	CovidXray [192]	Success	Failure
AlexNet [81]	0.9268	0.9738	0.8714	0.8526	0.9049	0.0951
ResNet [75]	0.9857	0.9832	0.9045	0.8990	0.9422	0.0578
VGG16 [98]	0.9785	0.9806	0.8501	0.8576	0.9145	0.0855
VGG19 [98]	0.9785	0.9811	0.8512	0.9279	0.9328	0.0672
Inception V3 [88]	0.9784	0.9879	0.8587	0.8998	0.9296	0.0704
SqueezeNet [184]	0.9756	0.9498	0.8288	0.8016	0.8858	0.1142
DenTnet [ours]	0.9928	0.9865	0.9157	0.8942	0.9463	0.0537

**Table 6:** PRS of various methods deeming four different datasets.

Models	PRS of various datasets				GMN of PRS	
	BreaKHis [33]	Malaria [191]	SkinCancer [193]	CovidXray [192]	Success	Failure
AlexNet [81]	0.9317	0.9656	0.8417	0.8744	0.9021	0.0979
ResNet [75]	0.9937	0.9793	0.9167	0.8667	0.9377	0.0623
VGG16 [98]	0.9936	0.9888	0.9055	0.8533	0.9334	0.0666
VGG19 [98]	0.9814	0.9753	0.8083	0.9872	0.9348	0.0652
Inception V3 [88]	0.9829	0.9713	0.8512	0.9796	0.9446	0.0554
SqueezeNet [184]	0.9854	0.9778	0.8871	0.7799	0.9036	0.0964
DenTnet [ours]	0.9700	0.9848	0.9258	0.8641	0.9350	0.0650

**Table 7:** RES of various methods deeming four different datasets.

Models	RES of various datasets				GMN of RES	
	BreaKHis [33]	Malaria [191]	SkinCancer [193]	CovidXray [192]	Success	Failure
AlexNet [81]	0.9647	0.9812	0.9154	0.8880	0.9366	0.0634
ResNet [75]	0.9854	0.9867	0.9010	0.9685	0.9597	0.0403
VGG16 [98]	0.9751	0.9718	0.8250	0.9846	0.9367	0.0633
VGG19 [98]	0.9875	0.9865	0.9065	0.9059	0.9457	0.0543
Inception V3 [88]	0.9854	0.9819	0.8874	0.9491	0.9501	0.0499
SqueezeNet [184]	0.9792	0.9197	0.7861	0.9514	0.9059	0.0941
DenTnet [ours]	0.9896	0.9879	0.9208	0.9629	0.9649	0.0351

**Table 8:** F1S of various methods deeming four different datasets.

Models	F1S of various datasets				GMN of F1S	
	BreaKHis [33]	Malaria [191]	SkinCancer [193]	CovidXray [192]	Success	Failure
AlexNet [81]	0.9479	0.9734	0.8770	0.8811	0.9189	0.0811
ResNet [75]	0.9896	0.9830	0.9129	0.9147	0.9494	0.0506
VGG16 [98]	0.9843	0.9803	0.8634	0.9143	0.9342	0.0658
VGG19 [98]	0.9845	0.9809	0.8546	0.9448	0.9397	0.0603
Inception V3 [88]	0.9844	0.9724	0.8693	0.9077	0.9322	0.0678
SqueezeNet [184]	0.9823	0.9479	0.8336	0.8571	0.9031	0.0969
DenTnet [ours]	0.9948	0.9864	0.9233	0.9108	0.9531	0.0469

**Table 9:** AUC of various methods deeming four different datasets.

Models	AUC of various datasets				GMN of AUC	
	BreaKHis [33]	Malaria [191]	SkinCancer [193]	CovidXray [192]	Success	Failure
AlexNet [81]	0.90	0.97	0.87	0.85	0.8964	0.1036
ResNet [75]	0.99	0.98	0.90	0.91	0.9441	0.0559
VGG16 [98]	0.98	0.98	0.86	0.85	0.9154	0.0846
VGG19 [98]	0.97	0.98	0.85	0.91	0.9260	0.0740
Inception V3 [88]	0.97	0.97	0.89	0.87	0.9239	0.0761
SqueezeNet [184]	0.97	0.95	0.83	0.75	0.8703	0.1297
DenTnet [ours]	0.99	0.99	0.91	0.90	0.9465	0.0535

**Table 10:** RTM of various methods deeming four different datasets.

Models	RTM in seconds of various datasets				GMN of RTM
	BreaKHis [33]	Malaria [191]	SkinCancer [193]	CovidXray [192]	
AlexNet [81]	07573	4100	1413	1328	2762.8
ResNet [75]	16889	3556	0799	2683	3368.5
VGG16 [98]	13419	7698	1450	1081	3567.2
VGG19 [98]	23502	7115	1255	1294	4059.4
Inception V3 [88]	14404	7357	1329	1189	3597.3
SqueezeNet [184]	20080	4140	1339	1864	3795.3
DenTnet [ours]	11083	7102	0873	1519	3196.3

**Table 11:** Summary of performance failure and RTM scores of miscellaneous deep learning algorithms.

Models	GMN scores of performance failure					GMN of RTM
	ACC	PRS	RES	F1S	AUC	
AlexNet [81]	0.0951	0.0979	0.0634	0.0811	0.1036	2762.8
ResNet [75]	0.0578	0.0623	0.0403	0.0506	0.0559	3368.5
VGG16 [98]	0.0855	0.0666	0.0633	0.0658	0.0846	3567.2
VGG19 [98]	0.0672	0.0652	0.0543	0.0603	0.0740	4059.4
Inception V3 [88]	0.0704	0.0554	0.0499	0.0678	0.0761	3597.3
SqueezeNet [184]	0.1142	0.0964	0.0941	0.0969	0.1297	3795.3
DenTnet [ours]	0.0537	0.0650	0.0351	0.0469	0.0535	3196.3

**Table 12:** Average ranking of each algorithm using nonparametric statistical tests. The best results are shown in bold.

Algorithms	Multiple comparison tests		
	Friedman ranking [196]	Friedman's aligned ranking [198]	Quade ranking [199]
AlexNet [81]	5.3333	26.0000	4.6189
ResNet [75]	2.1667	09.0000	2.2857
VGG16 [98]	4.6667	27.8333	4.6191
VGG19 [98]	4.0000	21.6667	4.3333
Inception V3 [88]	3.6667	22.1667	4.0952
SqueezeNet [184]	6.6667	36.6667	6.6667
DenTnet [ours]	**1.5000**	**07.1667**	**1.3809**
Various statistics	24.500000	23.102557	5.274194
*p* value	0.000422	0.000763	0.000820

**Table 13:** Results achieved on post hoc comparisons for adjusted *p* values, with *α*=0.05 and *α*=0.10.

Index	Algorithms	*p* values	*α*=0.05		*α*=0.10	
			Holm [202]	Shaffer [211]	Holm [202]	Shaffer [211]
1	VGG19 [98] versus Inception V3 [88]	0.789268	0.050000	0.050000	0.100000	0.100000
2	ResNet [75] versus DenTnet [ours]	0.592980	0.025000	0.025000	0.050000	0.050000
3	VGG16 [98] versus VGG19 [98]	0.592980	0.016667	0.016667	0.033333	0.033333
4	AlexNet [81] versus VGG16 [98]	0.592980	0.012500	0.016667	0.025000	0.033333
5	VGG16 [98] versus Inception V3 [88]	0.422678	0.010000	0.016667	0.020000	0.033333
6	AlexNet [81] versus SqueezeNet [184]	0.285049	0.008333	0.008333	0.016667	0.016667
7	AlexNet [81] versus VGG19 [98]	0.285049	0.007143	0.007143	0.014286	0.014286
8	ResNet [75] versus Inception V3 [88]	0.229102	0.006250	0.006250	0.012500	0.012500
9	AlexNet [81] versus Inception V3 [88]	0.181449	0.005556	0.005556	0.011111	0.011111
10	ResNet [75] versus VGG19 [98]	0.141579	0.005000	0.005000	0.010000	0.010000
11	VGG16 [98] versus SqueezeNet [184]	0.108809	0.004545	0.004545	0.009091	0.009091
12	Inception V3 [88] versus DenTnet [ours]	0.082352	0.004167	0.004167	0.008333	0.008333
13	VGG19 [98] versus DenTnet [ours]	0.045021	0.003846	0.003846	0.007692	0.007692
14	ResNet [75] versus VGG16 [98]	0.045021	0.003571	0.003571	0.007143	0.007143
15	VGG19 [98] versus SqueezeNet [184]	0.032509	0.003333	0.003333	0.006667	0.006667
16	Inception V3 [88] versus SqueezeNet [184]	0.016157	0.003125	0.003333	0.006250	0.006667
17	VGG16 [98] versus DenTnet [ours]	0.011118	0.002941	0.003333	0.005882	0.006667
18	AlexNet [81] versus ResNet [75]	0.011118	0.002778	0.003333	0.005556	0.006667
19	AlexNet [81] versus DenTnet [ours]	0.002116	0.002632	0.003333	0.005263	0.006667
20	ResNet [75] versus SqueezeNet [184]	0.000309	0.002500	0.003333	0.005000	0.006667
21	SqueezeNet [184] versus DenTnet [ours]	0.000034	0.002381	0.002381	0.004762	0.004762

**Table 14:** Adjusted *p* values for various tests considering DenTnet [ours] as control method.

Tests	Algorithms	Not	1 × *N* post hoc procedures and *p* values							
		adjusted	1-2 step-procedure		Step-down procedures			Step-up procedures		
		*p* values	*p*_*Bonf*_ [201]	*p*_*Li*_ [209]	*p*_*Holm*_ [202]	*p*_*Hol*_ [206]	*p*_*Finn*_ [208]	*p*_*Hoch*_ [203]	*p*_*Hom*_ [204]	*p*_*Rom*_ [207]
Friedman [196]	SqueezeNet [184]	0.000034	0.000206	0.000084	0.000206	0.000206	0.000206	0.000206	0.000206	0.000196
	AlexNet [81]	0.002116	0.012694	0.005171	0.010578	0.010533	0.006333	0.010578	0.010578	0.010060
	VGG16 [98]	0.011118	0.066705	0.026588	0.044470	0.043734	0.022112	0.044470	0.044470	0.042403
	VGG19 [98]	0.045021	0.270125	0.099595	0.135063	0.129073	0.066765	0.135063	0.123528	0.135063
	Inception V3 [88]	0.082352	0.494113	0.168281	0.164704	0.157923	0.097990	0.164704	0.164704	0.164704
	ResNet [75]	0.592980	3.557881	0.592980	0.592980	0.592980	0.592980	0.592980	0.59298	0.592980

F. al. rank [198]	SqueezeNet [184]	0.000031	0.000187	0.000152	0.000187	0.000187	0.000187	0.000187	0.000187	0.000178
	VGG16 [98]	0.003525	0.021147	0.016964	0.017623	0.017499	0.010536	0.017623	0.017623	0.016759
	AlexNet [81]	0.007837	0.047023	0.036954	0.031348	0.030982	0.015613	0.031348	0.031348	0.029891
	Inception V3 [88]	0.034193	0.205155	0.143404	0.102578	0.099110	0.050848	0.081277	0.068385	0.081277
	VGG19 [98]	0.040638	0.243830	0.165952	0.102578	0.099110	0.050848	0.081277	0.081277	0.081277
	ResNet [75]	0.795758	4.774545	0.795758	0.795758	0.795758	0.795758	0.795758	0.795758	0.795758

Quade [199]	SqueezeNet [184]	0.027879	0.167272	0.086779	0.167272	0.156038	0.156038	0.167272	0.167272	0.159049
	AlexNet [81]	0.177939	1.067632	0.377531	0.889693	0.624577	0.444463	0.517618	0.388213	0.517618
	VGG16 [98]	0.177939	1.067632	0.377531	0.889693	0.624577	0.444463	0.517618	0.388213	0.517618
	VGG19 [98]	0.219348	1.316086	0.427803	0.889693	0.624577	0.444463	0.517618	0.438695	0.517618
	Inception V3 [88]	0.258809	1.552853	0.468693	0.889693	0.624577	0.444463	0.517618	0.517618	0.517618
	ResNet [75]	0.706617	4.239701	0.706617	0.889693	0.706617	0.706617	0.706617	0.706617	0.706617

**Table 15:** Adjusted *p* values of tests for multiple comparisons among all methods.

Index	Hypothesis	*N* × *N* post hoc procedures and *p* values				
		Unadjusted	Nemenyi [210]	Holm [202]	Shaffer [211]	Bergmann [212]
1	SqueezeNet [184] versus DenTnet [ours]	0.000034	0.000721	0.000721	0.000721	0.000721
2	ResNet [75] versus SqueezeNet [184]	0.000309	0.006479	0.006171	0.004628	0.004628
3	AlexNet [81] versus DenTnet [ours]	0.002116	0.044428	0.040197	0.031734	0.031734
4	AlexNet [81] versus ResNet [75]	0.011118	0.233469	0.200116	0.166763	0.111176
5	VGG16 [98] versus DenTnet [ours]	0.011118	0.233469	0.200116	0.166763	0.122293
6	Inception V3 [88] versus SqueezeNet [184]	0.016157	0.339296	0.258511	0.242354	0.177726
7	VGG19 [98] versus SqueezeNet [184]	0.032509	0.682698	0.487642	0.487642	0.292585
8	ResNet [75] versus VGG16 [98]	0.045021	0.945439	0.630292	0.495230	0.315146
9	VGG19 [98] versus DenTnet [ours]	0.045021	0.945439	0.630292	0.495230	0.405188
10	Inception V3 [88] versus DenTnet [ours]	0.082352	1.729397	0.988227	0.905874	0.494113
11	VGG16 [98] versus SqueezeNet [184]	0.108809	2.284998	1.196904	1.196904	0.652857
12	ResNet [75] versus VGG19 [98]	0.141579	2.973156	1.415789	1.415789	0.652857
13	AlexNet [81] versus Inception V3 [88]	0.181449	3.810433	1.633043	1.633043	1.270144
14	ResNet [75] versus Inception V3 [88]	0.229102	4.811140	1.832815	1.633043	1.270144
15	AlexNet [81] versus VGG19 [98]	0.285049	5.986038	1.995346	1.995346	1.270144
16	AlexNet [81] versus SqueezeNet [184]	0.285049	5.986038	1.995346	1.995346	1.425247
17	VGG16 [98] versus Inception V3 [88]	0.422678	8.876240	2.113390	2.113390	1.690712
18	AlexNet [81] versus VGG16 [98]	0.592980	12.452582	2.371920	2.371920	1.778940
19	VGG16 [98] versus VGG19 [98]	0.592980	12.452582	2.371920	2.371920	1.778940
20	ResNet [75] versus DenTnet [ours]	0.592980	12.452582	2.371920	2.371920	1.778940
21	VGG19 [98] versus Inception V3 [88]	0.789268	16.574629	2.371920	2.371920	1.778940

## Data Availability

The four following publicly available datasets were used in this study: BreaKHis [33] (https://www.kaggle.com/datasets/ambarish/breakhis), Malaria [191] (https://www.kaggle.com/iarunava/cell-images-for-detecting-malaria), CovidXray [192] (https://github.com/ieee8023/covid-chestxray-dataset), and SkinCancer [193] (https://www.kaggle.com/fanconic/skin-cancer-malignant-vs-benign).

## Abbreviations

*BreaKHis*: Breast cancer histopathological image classification
*BACH*: Breast cancer histology images
*CNN*: Convolutional neural network
*DenseNet*: Dense convolutional Network
*ResNet*: Resi du al network
*VGG*: Visual geometry group at the University of Oxfor d
*DDSM*: Digital da tabase for screening mammography
*CBIS* − *DDSM*: Curate d breast imaging subset of *DDSM*
*SVM*: Support vector machine
*H*&*E*: Haematoxylin an d eosin
*BN*: Batch normalization
*ReLU*: Rectifie d linear unit
*ROC*: Receiver operating characteristic
*AUC*: Area un de r the ROC curve
*ACC*: Accuracy
*GMN*: Geometric mean
*PRS*: Precision score
*RES*: Recall score
*F*1*S*: *F*1 score
*RTM*: Runtime.
